The article "The Application of Internet of Things in Robot Route Planning Based on Multisource Information Fusion" was published in 2022. Journal: Comput Intell Neurosci.

# The Application of Internet of Things in Robot Route Planning Based on Multisource Information Fusion

**DOI:** 10.1155/2022/1707259

**Published:** 2022-06-17

**Authors:** Yunfeng Yao, Na He, Min Zhang

**Affiliations:** ^1^College of Mechanical and Electrical Engineering, Jiaxing Nanhu University, Jiaxing, Zhejiang 314001, China; ^2^Gongqing Institute of Science and Technology, Gongqingchengshi, Jiangxi 332020, China; ^3^Dean's Office of Henan Polytechnic University, Henan Polytechnic University, Jiaozuo, Henan 454000, China

## Abstract

With the advent of the Internet of Everything era, multi-information integration, and development, technology has penetrated into all aspects of life, promoting the continuous progress of social development, and people's requirements for a happy life are getting higher and higher. In this, robots play an extremely important role. It is especially important for the route planning of robots. This paper analyzes the DWA dynamic window algorithm through the verification of the global route planning algorithm, namely, the Dijkstra algorithm and the *A*^*∗*^ algorithm; the verification of the local route planning algorithm; the application of the DWA mobile robot algorithm in the robot route planning. The three aspects of the evaluation function are described by a formula, the experimental simulation is carried out, the relationship between the evaluation function terms is obtained, and the feasibility of the algorithm is verified.

## 1. Introduction

With the continuous progress of the times, the continuous development of science and technology, and the continuous improvement of people's living needs, the participation of robots in life is getting higher and higher, and the practical application scenarios of robots are becoming more and more extensive. It is a very obvious trend that the application scenarios of robots have begun to shift to the service industry on a large scale and are no longer limited to industrial production. This also means that the robot industry has become one of the important industries for China's future development and will play an important role in promoting China's industrial transformation and upgrading, and the replacement of labor by robots will also be the trend of future manufacturing.

Nowadays, all kinds of robots participate in various activities in people's social life, such as mobile robot [1], rehabilitation robot [2], lower limb robot [3], experimental quantitative robot [4], distributed multirobot [5], robot-assisted surgery [6]. These versatile robots not only replace people in repetitive and intensive manual labor but also greatly increase the efficiency of manufacturing, reduce labor costs, and play an important role in social development.

The article "The Application of Internet of Things in Robot Route Planning Based on Multisource Information Fusion" was published in 2022. Journal: Comput Intell Neurosci.

The route planning technology is one of the core contents of the research in the field of robotics, and the robot must navigate according to the planned path. Different types of robots adapt to different route planning. Path planning for transportation systems [7] can reduce hazards on turn-limited routes [8]. Multimodal transport route planning [9] integrates personalized route planning methods with different decision-making strategies [10] to solve the problem of optimizing the route planning of automatic guided vehicles (AGVs) in semiconductor manufacturing plants [11]. The comprehensive three-dimensional analysis of urban environment based on network [12] describes the road for strangers in the city, which requires completely different cognitive processes and strategies from the actual walking to the destination, and can highly adapt to the degree of perceptual information available for the task [13].

With the continuous development of communications, the Internet of Things [14] realized by the latest developments in RFID, smart sensors, communication technologies, and Internet protocols, as a belated communication worldview [15], is closely related to many fields [16]. The proposed information fusion method is applied to formation drill ability prediction [17], state of the art in robust speech processing [18], constraint fusion analysis [19], Bayesian network fault diagnosis method based on multisource information fusion [18, 20], and integrating a large number of different heterogeneous terminal systems to develop a large number of digital services [21]. Accompanying the rapid growth in the number of sensors deployed globally [22] is the discovery of services and on-demand provisioning of missing functions in an infrastructure consisting of a large number of networked, resource-constrained devices [23].

## 2. About the Theoretical Basis

### 2.1. Information Fusion

#### 2.1.1. Advantages and Applications of Multisource Information Fusion Technology

The sensor collects multiple information and confirms different sensor systems multiple times so as to improve the reliability and detection capability of the sensor system, improve the quality and credibility of the system detection data and information, improve the system's perception of specific data and the ability of data logical reasoning, speed up the accuracy and response speed of the system, and improve the detection reliability of the system. Data fusion of data information obtained by sensors from different information sources improves the system's information decision-making and analysis capabilities, shortens the system's information response delay time, and improves the system's information detection and processing performance. Information fusion processing is an information processing behavior that imitates biological environmental conditions. At the same time, information fusion processing can also be regarded as a comprehensive optimization process of information processing and multisource collection. Its purpose is to help people make accurate decisions and accurately judge the behavior of individuals or groups by optimizing information.

The article "The Application of Internet of Things in Robot Route Planning Based on Multisource Information Fusion" was published in 2022. Journal: Comput Intell Neurosci.

The most beneficial application of multisource information fusion is in medicine. On the one hand, it directly measures human physiological and medical data through multiple medical sensor probes and then simultaneously transmits it to the upper computer operation interface of patients, family members, and even doctors and community doctors. Based on the measured physiological and physical data, a conclusion is drawn whether the body meets the health standards. The physiological data and the measured waveform image data transmitted by the doctor through the probe can effectively and in real time help the patient determine the current user's physical health status, and the patient can also directly obtain information and results about their own health assessment; on the other hand, it is important to help patients retrieve similar symptoms and medical waveform images through medical waveform images and semantic information retrieval and to fuse semantic information with the current patient's situation, so as to help patients be diagnosed and treated in a timely manner and better prevent and treat various diseases. This not only greatly saves the time of seeing a patient but also reduces the cost of seeing a patient. In addition, it has made great contributions to the timely diagnosis of the early causes of cardiovascular diseases and other diseases and the early detection of clinical signs of the disease, which can effectively reduce the mortality rate of the disease.

#### 2.1.2. IoT Information Fusion

The Internet of Things is a new type of electronic technology or data network system developed on the basis of Internet technology. With the rapid development of the network and the progress of sensor networks, the research on the Internet of Things and its technology has become the future development direction of the Internet. This electronic technology or network system is mainly based on the coding of electronic products and uses RFID identification technology to identify and identify all physical items in the world so as to realize dynamic monitoring of physical items. Among them, digital calculation modules, data calculation, and so on will be used. In addition, purely technically speaking, the Internet of Things is an interconnected structure of things, objects, and intelligence about RFID technology, remote sensing technology, nanotechnology, and intelligent identification technology. Of course, the Internet of Things itself is also an expansion of Internet technology because the Internet of Things is mainly developed based on network technology and then controls physical objects on a larger scale. However, in the evolution and development, the Internet of Things is also a business or application, especially in today's society; in addition to technological innovation, the Internet of Things must continuously optimize its applications and develop the Internet of Things model based on user experience.

The article "The Application of Internet of Things in Robot Route Planning Based on Multisource Information Fusion" was published in 2022. Journal: Comput Intell Neurosci.

The Internet of Things information fusion technology refers to the analysis, refinement, and integration of information data obtained by sensors. The purpose of applying this technology is to obtain more accurate information data so as to provide information data for certain decision-making needs or data analysis. The key of information fusion technology is to refine the information data so as to improve the practicability of the information data. The main application field of information fusion technology is the military field, but it has gradually expanded to the civilian field and has played a huge role. According to the different levels of information and data fusion, IoT information fusion technology can be divided into three levels: data-level fusion technology, feature-level fusion technology, and decision-level fusion technology.

### 2.2. Robot

Since the 1950s, many countries in the world have vigorously developed the robot industry. Americans were the first to research and develop the first industrial application robot. The role of this robot is to replace people in repetitive and intensive manual labor, which greatly increases the efficiency of manufacturing and reduces labor costs. The development of robots is the result of the development of human society and science and technology. On the one hand, the development of robots has a significant impact on human society. Robots are typical representatives of high-end intelligent equipment and core assets. From a national perspective, robot technology is even an important factor in examining a country's technological level and technological innovation capabilities. Therefore, many countries in the world have long paid special attention to the development of robots, and some countries have even raised the development of robots to the height of the national scientific and technological strategic layout and successively introduced a series of related measures to encourage and stimulate the development of the robot industry. In the layout plan of “Made in China 2025” proposed by my country in 2015, the development of robots has been raised to a national strategic perspective. Government departments have released a series of relevant measures for the development of robots. Robots have received unprecedented development opportunities. A large number of robots have gradually become a reality and have been applied to all walks of life. At the same time, the functions of robots are becoming more and more powerful and meet people's needs.

The article "The Application of Internet of Things in Robot Route Planning Based on Multisource Information Fusion" was published in 2022. Journal: Comput Intell Neurosci.

In recent years, the practical application scenarios of robots have become more and more extensive. It is a very obvious trend that the application scenarios of robots have begun to shift to the service industry on a large scale and are no longer limited to industrial production. Especially in this year's fight against the epidemic, service robots have played a huge role. Service robots have been quickly put into the fight against the epidemic. They can automatically detect the body temperature of passing people and perform disinfection and sterilization functions in public places, greatly reducing the work pressure of epidemic prevention personnel. Reflecting the superiority of service robots, it is a temperature measurement and disinfection robot.

Service robots have entered an unstoppable trend from public service places to home applications. One of the important reasons is that the aging problem in some developed countries in the world is already very serious. The reality makes the pension problem even more serious: on the one hand, because the pace of modern life has been accelerating, young people are facing huge work challenges and do not have more energy to accompany the elderly at home and take care of housework. The cost of the elderly has increased significantly. In the case of increasing aging, there will be a reality that there is no ability to take good care of the elderly and ensure a better life for the elderly. This is not only an urgent problem for a family but also an urgent problem for society.

#### 2.2.1. Development and Research Status of Robots

Entering the 21st century, with the continuous development of the economy and society, the domestic economy is changing from a labor-intensive manufacturing method to an increasing demand for automated robots to replace manual labor. The reason for this is that the labor-intensive and extensive manufacturing pattern in the country in the past few decades was difficult to maintain due to the declining demographic dividend of the aging population. The robot industry has become one of the important industries for China's future development and will play an important role in promoting China's industrial transformation and upgrading, and the replacement of labor by robots will also be the trend of future manufacturing.

The article "The Application of Internet of Things in Robot Route Planning Based on Multisource Information Fusion" was published in 2022. Journal: Comput Intell Neurosci.

With the continuous development of robots, more and more disciplines are covered. In addition to traditional electronic information, mechanical design, sensor technology, information processing, and computers, more and more bioelectric signals, material design, nanotechnology, and so on are involved. Intelligence is also progressing. Robots are widely used in industry. In addition, the application of robots in other work environments that are difficult for humans to reach and to meet the specific requirements of people in specific situations, such as service fields and military fields, is also extremely important. The most popular robot recently is the robot dog made by Boston Dynamics Engineering Company for the military. It is used for tasks such as transporting materials in rugged mountains during wartime. It has a vision system that can be used to perform related tasks autonomously and has a certain intelligence. Different from the previous way of walking on wheels, Big Dog adopts a bionic limb design and is equipped with four legs to walk, which can climb, jump, and resist side impact.

#### 2.2.2. Classification of Robots

Robots have gradually become a research hotspot of artificial intelligence and have developed rapidly. Robots are mainly divided into aerial drones and ground mobile robots. UAVs are widely used in logistics and distribution, fire warning, target detection, border patrol, and so on. However, due to the limited endurance of the UAV, it can only work continuously for 20–30 minutes before replacing the battery, making it unable to perform time-consuming tasks, and its load capacity is limited, thus limiting the development of UAVs. Mobile robots have large loads and can perform tasks for a long time.

With the development of science and technology and the emergence of various complex environments and complex tasks, it is difficult for a single robot to meet the requirements of more and more complex tasks, especially in the military, police departments, logistics distribution, and other industries. The task execution efficiency of a single flying robot is low, and multirobot cooperation is needed. There are three main types of multirobots: multi-UAV, multimobile robot, and heterogeneous robot system composed of UAV and mobile robots. Among them, due to the respective advantages of drones and mobile robots, the combination of drones and mobile robots makes up for the shortcomings of short battery life and limited load when drones work alone and at the same time makes up for the lack of wide vision of mobile robots. The disadvantage of not being flexible enough to exercise, combining the advantages of the two, has the advantages of time, space, and function. Heterogeneous robot systems can adapt to more and more complex task requirements and have broad application prospects in military, agriculture, industry, and service industries.

The article "The Application of Internet of Things in Robot Route Planning Based on Multisource Information Fusion" was published in 2022. Journal: Comput Intell Neurosci.

## 3. Route Planning

Route planning technology is one of the core contents of the research in the field of robotics, and the robot navigates according to the route planning. The route planning of the robot can be divided into the robot moves from the starting position to the specified position; the algorithm can bypass the obstacles on the walking route during the movement of the robot, and at the same time, it can complete the specified work task in a specific position; based on the implementation of the first two problems, we try to optimize the walking route.

### 3.1. Classification of Planning Algorithms

The path planning of the robot is the problem of optimal path selection. Route planning algorithms can be generally classified according to different algorithm sources, whether it is a single algorithm to realize the path planning function, whether it is inspired by biology, whether it is a pure mathematical theory, and so on, as shown in Figure 1.

#### 3.1.1. Sampling-Based Methods

The core of the sampling-based path planning algorithm is to collect the environmental information of the space through sensors and then randomly sample the points in the space that are not within the obstacle range and connect the random sample points to form a path that can connect the beginning and end states to navigate. Since the algorithm only focuses on the points in the unobstructed space and does not process the obstacle points in the state space, it saves a lot of computing time. The algorithm does not construct the obstacle space. When there are too few sampling points or the distribution is not balanced, it will cause incompleteness. For example, Voronoi can perform global or local map planning; RRT is a fast path search without collision; PRM is a method based on graph search, which has the characteristics of complete probability and is not optimal.

#### 3.1.2. Algorithms of Mathematical Models and Multifusion Algorithms

The core idea of the algorithm of the mathematical model is to describe the motion state and constraint conditions in the form of mathematical optimization, and the representative algorithms include MILP and NLP.

The multifusion algorithm can realize the optimal solution of path planning. If a single algorithm may focus on fastness or effectiveness, the collective algorithm has better time performance and work effect than a single algorithm because it integrates multiple algorithms and integrates the advantages of multiple algorithms. A good advantage is the ability to achieve global optimization and cost minimization.

The article "The Application of Internet of Things in Robot Route Planning Based on Multisource Information Fusion" was published in 2022. Journal: Comput Intell Neurosci.

#### 3.1.3. Algorithms Based on Biological Heuristics

Bioinspired algorithms refer to researchers who, inspired by a phenomenon in the real natural environment, propose mathematical theories with similar ideas to solve some problems. There are three common algorithms.

Neural networks are widely used in pattern classification and other problems, using neurons to approximate any nonlinear function, and neural networks also have some related applications in path planning. The aspect of supervised learning is path planning with CNN's laser and A^*∗*^. The other is based on reinforcement learning. Given a planned goal, the machine can collide and update the network autonomously without the need to manually set a route.

The ant colony algorithm is a global algorithm, emphasizing the cooperation of individuals in the community. If the map is in grid format, and the ant colony algorithm is used in the grid map, the robot planning route will bring problems such as many turns and delays. The shortest path of each iteration needs to be further improved to achieve a more optimal path and real-time performance.

The genetic algorithm takes a single point in the whole space as an object and uses the probability method to search the space. Mathematically, it does not require the processing of structural objects required for function derivation and continuity; it can search the space by itself and plan the direction by itself. It has good global planning ability and strong robustness.

#### 3.1.4. Node-Based Approach

The node-based method is the grid method, which is used in grid maps. The grid map divides the spatial environment into the form of grids, in which each grid represents the probability of possession. The type of map used in the ROS system is a grid map. In raster maps, Dijkstra's algorithm and *A*^*∗*^ algorithm can be used as global static navigation algorithms; *D*^*∗*^ algorithm used in dynamic environments can also work well in changing environments.

### 3.2. Global Route Planning Algorithm

Global path planning is to search for an optimal or approximately optimal line that meets the conditions in all state spaces according to the constraints when the robot has obtained the position information of the objects in the space. In the grid method, the size of the divided grid needs to be based on the size of the robot so that the robot can use the global search optimization algorithm for path walking when navigating. The research of this subject is global route planning based on the grid method.

The article "The Application of Internet of Things in Robot Route Planning Based on Multisource Information Fusion" was published in 2022. Journal: Comput Intell Neurosci.

#### 3.2.1. Dijkstra Algorithm

Dijkstra's algorithm process is as follows:

1. Initially, *S*={*v*}, where the distance of *v* is 0. *Z* contains all vertices of the complement except *v*, *v*.
2. Select *d* with the smallest distance from *v* in *Z* and add it to *S*.
3. Using the newly added point *d* as the intermediate point, modify the distance of each vertex in *Z*. If the distance from point *v* to *Z* through *d* is shorter than the distance without *d*, then the *d* value of the vertex plus the weight is used as the new value of *Z*. Repeat steps 2 and 3 until the vertex set in *Z* is empty.

Dijkstra's algorithm is a greedy strategy. The algorithm compares and calculates from a global perspective to obtain the shortest path. Therefore, the maximum complexity of the algorithm is *O*(*n*^2^). When the number of nodes in a graph increases, the algorithm needs more time to calculate the weight comparison between nodes, resulting in the low efficiency of the algorithm. At the same time, due to the increase in the amount of calculation, the more the data that needs to be accessed, the larger the memory space occupied, and the certain requirements for the performance of the processor can better achieve the real-time effect.

#### 3.2.2. *A*^*∗*^ Algorithm

The *A*^*∗*^ algorithm is the global shortest path search algorithm. It is different from the Dijkstra algorithm's nondirectional diffusion method in the process of tracing. The *A*^*∗*^ algorithm is to search for the path directional toward the endpoint according to a certain cost function. The difference between the *A*^*∗*^ algorithm and the Dijkstra algorithm is also an improvement. Compared with the greedy strategy of Dijkstra's algorithm, which searches all over the space, the *A*^*∗*^ algorithm has a directional strategy, which needs to traverse relatively fewer nodes, and the search efficiency is higher. When the *A*^*∗*^ algorithm searches toward the endpoint, the evaluation function needs to be used to evaluate whether the route through the node to the endpoint is the optimal path. Different trajectories can be obtained according to the different evaluation functions used in the algorithm. The key evaluation function of the *A*^*∗*^ algorithm is

(1) $$\begin{array}{c} f\left(n\right)=g\left(n\right)+h\left(n\right). \end{array}$$

In the formula, *f*(*n*) represents the total evaluation function of the current node *n*; *g*(*n*) represents the actual cost from the starting point to the current point; *h*(*n*) represents the estimated cost from the current node to the endpoint.

The article "The Application of Internet of Things in Robot Route Planning Based on Multisource Information Fusion" was published in 2022. Journal: Comput Intell Neurosci.

The value of *h*(*n*) determines the performance of the algorithm. *h*(*n*) often uses Euclidean distance and Manhattan distance as the value of the algorithm for two points in space. By using the Manhattan distance as the value of *h*(*n*), there are two points (*X*_1_, *Y*_1_)  and (*X*_2_, *Y*_2_):

(2) $$\begin{array}{c} D_{\text{Manhattan}}=\left|x_{1}-x_{2}\right|+\left|y_{1}-y_{2}\right|. \end{array}$$

### 3.3. Local Route Planning Algorithm

In the actual environment, the robot cannot safely reach the designated position strictly according to the established path due to the inaccuracy of the actual measurement information and the change of the environment due to the accuracy of its own sensor. The global application is used in static planning, and local path planning is required in dynamic planning. In the local path planning algorithm, the robot continuously collects the position information of the surrounding obstacles through the sensor during the walking process and at the same time predicts the obstacle information on the original map in advance so as to realize the local dynamic planning and make it conform to the previous global plan. The DWA dynamic window method performs multiple sets of velocity sampling within the window range to simulate the planned path; the artificial potential field method is to construct a virtual artificial potential field in space. For a single local planning algorithm, the robot has high real-time performance and good practicability in the process of path planning. However, if there is no global reference information, the robot is prone to fall into local extreme points, causing the robot to fail to reach the target point according to the instructions. For this reason, it is necessary to match the global planning while applying the local planning algorithm so as to better ensure that the robot navigates to the specified target position normally.

#### 3.3.1. DWA Mobile Robot Algorithm

The dynamic window method (DWA) is mainly used in indoor static environments. Local path planning is performed with the assistance of paths planned with the help of a global algorithm. Its core is to continuously collect its own robot pose and external environment information through the measurement sensor carried within a certain time interval and obtain a series of acceleration and angular velocity by sampling. Because the sampled acceleration and angular velocity are within a range of values, it is called a window, and the sampled acceleration and angular velocity are used to numerically simulate the path that the robot will walk. Multiple paths can be obtained through numerical calculation and simulation, and then the optimal path is selected relative to the current motion control variables of the robot according to the evaluation function used as the basis for the selection of the scheme.

The article "The Application of Internet of Things in Robot Route Planning Based on Multisource Information Fusion" was published in 2022. Journal: Comput Intell Neurosci.

The DWA algorithm needs to obtain the model state expression of the robot. Therefore, a two-wheeled robot based on differential drive has no velocity in the *y*-axis direction. And the motion trajectory of the robot in two sampling adjacent periods can be approximately considered as a straight line. Assuming that the robot travels a small distance at an angle *θt* between the speed *v* and the *x*-axis during the Δ*t* time, the movement increments Δ*x* and Δ*y* of the robot on the *x*-axis and the *y*-axis can be obtained:

(3) $$\begin{array}{c} \Delta x=x+v\Delta t\;\cos\left(\theta t\right),\\ \Delta y=y+v\Delta t\;\sin\left(\theta t\right). \end{array}$$

From the above, the mathematical expression of the moving mathematical trajectory is as follows:

(4) $$\begin{array}{c} x=x+v\Delta t\;\cos\left(\theta t\right),\\ y=y+v\Delta t\;\sin\left(\theta t\right),\\ \theta t=\theta t+w\Delta t. \end{array}$$

During the sampling of the speed window, the robot body collects multiple sets of trajectory speed values. In order for the robot to safely perform path planning within the tolerance range of its own control performance, some necessary speed limits are required. During operation, the robot first performs a limited range of speed and angular velocity value changes, and the range formula is as follows:

(5) $$\begin{array}{c} V_{m}=\left\{v\in \left[v_{\text{min}},v_{\text{max}}\right],w\in \left[w_{\text{min}},w_{\text{max}}\right]\right\}. \end{array}$$

And because the robot has different torque performance parameters when selecting the motor, the robot starts from the angle of the motor. Knowing the current speed *v*_*c*_ and angular speed *w*_*c*_ of the robot at this moment, it must also satisfy the actual speed that can be achieved:

(6) $$\begin{array}{c} V_{d}=\left\{\left(v,w\right)|v\in \left(v_{c}-{\dot{\nu }}_{b}\Delta t,v_{c}+{\dot{\nu }}_{a}\Delta t\right),w\in \left(w_{c}-{\dot{w}}_{b}\Delta t,w_{c}+{\dot{w}}_{a}\Delta t\right)\right\}. \end{array}$$

In the formula, ${\dot{\nu }}_{a}$ and ${\dot{w}}_{a}$ are the maximum acceleration; ${\dot{\nu }}_{b}$ and ${\dot{w}}_{b}$ are the maximum deceleration.

Finally, when the robot can safely detour when it encounters obstacles during walking, the following formula for the speed needs to be satisfied within the range of the speed value:

(7) $$\begin{array}{c} V_{d}=\left\{\left(v,w\right)|v_{c}\leq \sqrt{2\cdot \text{dis}\left(v.w\right)\cdot {\dot{\nu }}_{b}},w_{c}\leq \sqrt{2\cdot \text{dis}\left(v.w\right)\cdot {\dot{w}}_{b}}\right\}. \end{array}$$

In the formula, dis(*v*.*w*) is the minimum distance of obstacles on the planned trajectory.

The article "The Application of Internet of Things in Robot Route Planning Based on Multisource Information Fusion" was published in 2022. Journal: Comput Intell Neurosci.

On the basis of the trajectory that meets the speed requirements, the evaluation function is used to evaluate, and the optimal trajectory is selected:

(8) $$\begin{array}{c} G\left(v,w\right)=\sigma \left(\alpha \text{head}\left(v,w\right)\right)+\beta \text{dis}\left(v,w\right)+\gamma \text{vel}\left(v,w\right). \end{array}$$

Among them, *α*head(*v*, *w*) represents the gap between the target angle of the assessment and the end of the route; dis(*v*, *w*) is the minimum distance of obstacles on the planned route; vel(*v*, *w*) represents the speed evaluation at this moment; *σ* is a smooth function; and *α*, *β*, and *γ* are evaluation coefficients.

### 3.4. Mathematical Theory of Graph Optimization

Graph optimization is expressed in the form of a graph according to the relationship between points and edges. When using the optimization algorithm in SLAM, the key is to describe the nonlinear motion state estimation of the robot in the form of a graph to optimize the solution. The robot can obtain an observation data *z*_*i*_ of the position at the position *x*_*i*_ at each moment through the sensor carried by itself. For this reason, it can be expressed by a functional relationship:

(9) $$\begin{array}{c} z_{i}=h\left(x_{i}\right). \end{array}$$

Since the data is collected by the robot's own sensor, there must be noise. For this reason, there are error terms on both sides of the above formula. The error terms of the observation equation of the robot are defined as follows:

(10) $$\begin{array}{c} e_{i}=z_{i}-h\left(x_{i}\right). \end{array}$$

In the robot, the graph model obtained from the robot's pose and observation point has *n* edges, and the optimized objective function can be obtained:

(11) $$\begin{array}{c} \underset{x}{\min}\sum_{i=1}^{n}e_{i}{\left(x_{i},z_{i}\right)}^{T}\Omega_{i}e_{i}\left(x_{i},z_{i}\right), \end{array}$$

where *z*_*i*_ is the observation data, *x*_*i*_ is the observation point, and Ω_*i*_ is the inverse of the covariance matrix.

Since the observation data *z*_*i*_ is the data collected by the robot at each sampling point, it can be obtained directly. Therefore, the objective function can be simplified and written in the form of the following sum:

(12) $$\begin{array}{c} \min F\left(x\right)=\sum_{i=1}^{n}e_{k}{\left(x_{i}\right)}^{T}\Omega_{i}e_{i}\left(x_{i}\right). \end{array}$$

From the optimization function obtained above, since the robot has multiple edges and multiple nodes in the actual operation process, when our goal is to solve it, we only need to get one of the initial points and the iteration direction. When only one edge is considered and an increment Δ*x* is calculated for the initial point ${\tilde{x}}_{i}$, the error term becomes $e_{i}\left({\tilde{x}}_{i}+\Delta x\right)$, and the first-order Taylor expansion can be obtained:

(13) $$\begin{array}{c} e_{i}\left({\tilde{x}}_{i}+\Delta x\right)\approx e_{i}\left({\tilde{x}}_{i}\right)+\frac{\text{d}e_{i}}{\text{d}x_{i}}\Delta x,\\ e_{i}\left({\tilde{x}}_{i}+\Delta x\right)=e_{i}+J_{i}\Delta x. \end{array}$$

Among them, *J*_*i*_ is the derivative of *e*_*i*_ with respect to *x*_*i*_:

(14) $$\begin{array}{c} J_{i}=\frac{\text{d}e_{i}}{\text{d}x_{i}}. \end{array}$$

It can be obtained by the formula, and the following formula can be obtained for the objective function of the *i*-th edge:

(15) $$\begin{array}{c} F_{i}\left({\tilde{x}}_{i}+\Delta x\right)=e_{i}{\left({\tilde{x}}_{i}+\Delta x\right)}^{T}\Omega_{i}e_{i}\left({\tilde{x}}_{i}+\Delta x\right),\\ F_{i}\left({\tilde{x}}_{i}+\Delta x\right)\approx {\left(e_{i}+J_{i}\Delta x\right)}^{T}\Omega_{i}\left(e_{i}+J_{i}\Delta x\right),\\ F_{i}\left({\tilde{x}}_{i}+\Delta x\right)=e_{i}^{T}\Omega_{i}e_{i}+2e_{i}^{T}\Omega_{i}J_{i}\Delta x+\Delta x^{T}J_{i}^{T}\Omega_{i}J_{i}\Delta x,\\ F_{i}\left({\tilde{x}}_{i}+\Delta x\right)=C_{i}+2b_{i}\Delta x+\Delta x^{T}H_{i}\Delta x. \end{array}$$

In the formula, *C*_*i*_ is the integration of terms unrelated to Δ*x*; 2*b*_*i*_ is the coefficient of the first-order term; *H*_*i*_ is the coefficient of the quadratic term.

The article "The Application of Internet of Things in Robot Route Planning Based on Multisource Information Fusion" was published in 2022. Journal: Comput Intell Neurosci.

In the above formula, since *C*_*i*_ is an item unrelated to Δ*x*, it is simplified and solved, and when all edges in the SLAM graph model are considered, all edges can be obtained by removing the subscripts of the parameters, and then the incremental equation can be obtained:

(16) $$\begin{array}{c} H\Delta x=-b. \end{array}$$

When the robot model is running, the number of edges constituting the graph is huge, and there are many parameters to be solved, but it is sparse, so it is possible to solve it in real time.

The graph-optimized SLAM algorithm, that is, the core formula of Hector SLAM, is solved by the Gauss–Newton method. The formula is as follows:

(17) $$\begin{array}{c} \varepsilon^{*}=\text{arg}\underset{\varepsilon }{\min}\sum_{i=1}^{n}{\left[1-M\left(s_{i}\left(\varepsilon \right)\right)\right]}^{2}. \end{array}$$

In the formula, *M*(*s*_*i*_(*ε*)) represents the map value corresponding to the grid under the point; *s*_*i*_(*ε*) represents the world coordinate corresponding to the laser point coordinate.

Based on the filtered SLAM, the particle filter algorithm formula is as follows:

(18) $$\begin{array}{c} P\left(x_{1:t},m|z_{1:t},u_{1:t-1}\right)=p\left(m|x_{1:t},z_{1:t}\right)\cdot p\left(x_{1:t}|z_{1:t},u_{1:t-1}\right), \end{array}$$

where *m* is the map, *u*_1:*t*−1_ is the chronometer data, *x*_1:*t*_ is the robot path, and *z*_1:*t*_ is the observation.

The article "The Application of Internet of Things in Robot Route Planning Based on Multisource Information Fusion" was published in 2022. Journal: Comput Intell Neurosci.

## 4. Validation Experiment

### 4.1. Dijkstra Algorithm Simulation Verification Experiment

Through the dynamic simulation experiment of the Dijkstra algorithm, one has the following:

1. By creating a 10 × 10 grid map as the search workspace, the red square is the starting point of the search, the green square is the end point of the search, and the black square represents obstacles.
2. Select the dark red square point as the search point, select four points from the minimum path of the dark red square to join the search range, the wine red square point is the point that has been searched, and the blue square point is the next step to be search point.
3. Repeat step (2) continuously, finally, search the square of the green endpoint, and the green route connecting the red start point and the green endpoint is the searched path.

Figure 2 shows the tracing process of Dijkstra's algorithm.  Figure 2(a), process 1, is the established 10 × 10 grid map, and the dark red starting point is used as the search center to find its four neighbors up, down, left, and right, making it blue. The color indicates the center to be searched next time, as shown in the second process of 2(b) in the figure, and calculates the distance from them to the starting point; in the third process of 2(c) in the figure, the point to the left of the dark red origin is taken as the new search starting point, the neighbor of the point is changed to blue, the distance from the new neighbor to the origin is calculated at the same time, and finally, the point to the left of the dark red origin is changed to wine red, indicating that the point has been searched. Through continuous outward diffusion, the steps shown in 2(d), process 4, are continuously cycled until the planned green path is found, as shown in 2(f), process 6.

### 4.2. *A*^*∗*^ Algorithm Simulation Verification Experiment

Using the same map as Dijkstra's algorithm in the previous section, the *A*^*∗*^ algorithm is dynamically simulated to evaluate its performance. The figure shows the tracing process of the *A*^*∗*^ algorithm. Unlike the Dijkstra algorithm, which has the characteristics of nondirectional outward diffusion at the closest distance to the origin, the *A*^*∗*^ algorithm uses the evaluation function to select the nearest neighbor to the endpoint as the center of the next search.

Comparing the path planning process of the *A*^*∗*^ algorithm in Figure 3 and the path planning process of the Dijkstra algorithm in Figure 2, it can be seen that, in the second process 3(b) of the figure in the initial stage, the execution process of the algorithm is the same as that of the Dijkstra algorithm. However, with the execution of algorithm *A*^*∗*^, the algorithm path begins to step in the direction of the upper right corner under the action of the formula evaluation function until it encounters an obstacle and starts to search up and down, and finally, the searched path is obtained. From the number of grids occupied by blue and red, the time efficiency of *A*^*∗*^ algorithm is better than that of the Dijkstra algorithm under this simulation condition.

The article "The Application of Internet of Things in Robot Route Planning Based on Multisource Information Fusion" was published in 2022. Journal: Comput Intell Neurosci.

### 4.3. DWA Algorithm Simulation Verification Experiment

Through the dynamic simulation of the DWA algorithm, the flowchart of the working effect of the algorithm is verified. In the simulation experiment, the value of the coefficient of the evaluation functions *α*=0.04, *β*=0.3, and *γ*=0.2 is shown in Figure 4 for the dynamic simulation result of the DWA algorithm. Figure 4(a) represents the obstacle, Figure 4(b) represents the navigation endpoint, Figure 4(c) represents the planned trajectory, and Figure 4(d) green represents the estimated trajectory sampled at different speeds.

When zooming in on the figure, you can see that the trajectory results of the velocity sampling are shown in Figure 5 in a window.

The optimal path is selected through the evaluation function after the sampling of multiple groups of speed. In the simulation process, it can be seen that when the current position of the robot is closer to the obstacle, the smaller dis(*v*.*w*) is, the slower the speed of the robot becomes, which causes *G*(*v*, *w*) to become smaller; on the contrary, the farther the distance is, the larger *C* is, and the speed of the robot also changes. The faster you go, the bigger *G*(*v*, *w*) becomes. It can be verified that the DWA algorithm can well complete the dynamic obstacle avoidance task so that the robot can safely reach the target point.

## 5. Conclusion

The path planning algorithm is the key for the robot to move to the target position accurately in the space environment. This paper introduces and compares the path planning algorithm of the robot, that is, the verification of the Dijkstra algorithm and the algorithm in the global route planning algorithm. Validation of the DWA mobile robot algorithm in planning algorithm in robot route planning. By comparing the two algorithms of global planning, the verification experiment shows that the time efficiency of the *A*^*∗*^ algorithm is better than that of the Dijkstra algorithm, and the DWA algorithm is verified to be able to complete the dynamic obstacle avoidance task well so that the robot can safely reach the target point. By analyzing and analyzing the DWA dynamic window algorithm, it is described by the formula from the three aspects of the motion model, speed sampling, and evaluation function, experimental simulation is carried out, the relationship between the evaluation function terms is obtained, and the feasibility of the algorithm is verified.

The article "The Application of Internet of Things in Robot Route Planning Based on Multisource Information Fusion" was published in 2022. Journal: Comput Intell Neurosci.

## Figures and Tables

**Figure 1:** Route planning classification.

**Figure 2:** Dijkstra's algorithm path planning process. (a) Process one. (b) Process two. (c) Process three. (d) Process four. (e) Process five. (f) Process six.

**Figure 3:** *A* ^*∗*^ algorithm path planning process. (a) Process one. (b) Process two. (c) Process three. (d) Process four. (e) Process five. (f) Process six.

**Figure 4:** DWA algorithm path planning process.

**Figure 5:** Speed sampling example.

## Data Availability

The experimental data used to support the findings of this study are available from the corresponding author upon request.
